# Multitask Learning with Graph Neural Network for Travel Time Estimation

**DOI:** 10.1155/2022/6622734

**Published:** 2022-03-28

**Authors:** Ling Yang, Shouxu Jiang, Fusheng Zhang

**Affiliations:** ^1^Faculty of Computing, Harbin Institute of Technology, Harbin 150006, Heilongjiang, China; ^2^Key Laboratory of Elevator Intelligent Safety in Jiangsu Province, Changshu Institute of Technology, Changshu 215500, Jiangsu, China

## Abstract

Travel time estimation (TTE) is widely applied for ride dispatching, ride-hailing, and route navigation. Even for a given trajectory, the travel time is affected by many spatial-temporal factors, including static ones such as distance, road type, and so on and dynamic ones such as speed, traffic condition, and so on. Challenges of accurate estimation lie in proper representation of these spatial-temporal factors and more importantly capturing the complex relationship among them for TTE. To tackle such challenges, we present a framework based on the fact that the travel time of each road segment is affected by its adjacent segments. It features a graph convolutional neural network and a recurrent neural network for basic TTE for each road segment and a graph attention network for the relation to estimations on the adjacent road segments. Finally, a multitask learning model is proposed for the travel time of the entire given path and that for each road segment. Experimental results on real taxi trajectory datasets of two cities show that the percentage estimation error of the new approach is well controlled at 13.91% and the proposed method outperforms three state-of-the-art methods significantly.

## 1. Introduction

Travel time estimation (TTE) is a classic yet challenging problem using trajectory data. In urban cities, it plays a key role in route planning [1], vehicle dispatching [2], and ride-hailing [3] applications, such as Uber, Lyft, and DiDi. The accuracy of TTE is vital to user stickiness and activity. According to [4], inaccurate travel time estimation leads to 28.4% car-booking cancellation.

There exist many factors that affect the accuracy of TTE, which can be summarized into two categories: the static ones such as road type, e.g., highway or byway, road width, speed limit, and in-degree and out-degree, and the dynamic ones such as weather, accident, traffic speed, time interval, and so on. It is worth noting that factors of road segments may have implicit dependency, which will affect TTE in a very complex way. For example, the speed on a road segment may be affected by its adjacent and congested segment since the vehicles have to slow down and wait.

To accurately estimate the travel time, such factors should be combined all together; however, there are three challenges to do so. (1) How to investigate the effects of these factors on the travel time, e.g., how does road type (e.g., main road and secondary road) affect the estimation of the travel time. (2) How to encode the complex factors and learn effective features from them, especially for the implicit ones, such as the traffic condition characteristics. Inadequate understanding of these factors may cause inaccuracy in the estimation. (3) How to fuse spatial-temporal correlation factors for travel time estimation. Among all these factors, traffic condition is the most important. Existing work on TTE [5–9] mainly aims to estimate the travel time of a path considering the factors such as traffic flow, weather condition, road type, and so on but lacks the study of the aforementioned implicit dependency among road segments.

To address the challenges, we present dependent relationship travel time estimation (DRTTE). We first analyze the relationship among various factors that may affect the estimation of the travel time. Based on the analysis, we then learn several features for TTE via a sequence of graph neural networks. We use graph convolutional network (GCN) to obtain spatial feature, followed by gated recurrent unit (GRU) capturing the spatial-temporal feature. The extracted features, when combined with auxiliary information, such as weather, are used to learn the traffic condition representation. The traffic condition representation, along with the road segment information, generates a vector for the speed on each road segment. Graph attention network (GAT) is then applied to update the speed vector considering the dependency of the road segments. With a multitask learning model, these new speed vectors are used in the final step for travel time estimation over all road segments and the entire path.

We highlight the following contributions in this work:

- Learning the road segment traffic conditions by exploring the static and the dynamic features.
- Proposing a multitask learning framework for learning the feature of each factor by exploiting the dependency and fusing them together to predict the travel time.
- Conducting extensive experiments to confirm the effectiveness of our proposed solution in comparison with the state-of-the-art baselines.

The rest of the paper is structured as follows. State-of-the-art solutions for TTE and related deep learning algorithms are reviewed in Section 2. The problem statement is given in Section 3. The methodology and computational framework are described in Section 4 and evaluated in Section 5. Finally, conclusions and discussions are given in Section 6.

## 2. Related Work

Machine learning and deep learning have been widely applied for spatial-temporal problems, including path inference [10], path query [11], path selection [12–14], crowd-sourcing analysis [15, 16], path traffic [5, 17], and travel time estimation. However, the above work aims to infer, query, or select a path, and less attention is paid on estimating the travel time which depends on relationship of road segments. Our method focuses on the two places: each road segment and the whole path. The SOTA methods focus on the whole path. In recent years, there are also many new approaches towards TTE. New methods of machine learning encoding the spatial-temporal features have been applied to solve TTE problems. ConLSTM [18] combined CNN and LSTM. Paper, [7, 9] proposed a data-driven regression model considering complex factors. DEEPTRAVEL [9] extracted multiple features of TTE for a path. Paper, [6, 19] utilized only GPS data for TTE. However, limitations such as path scale, auxiliary information, correlation, and dependency among road segments are not well addressed, leading to affected degree of accuracy.

## 3. Preliminary

### 3.1. Definitions

**Definition 1 .**

(directed graph for road network). A road network is represented as a directed graph *𝒢*=(*V*, *E*, **A**), where *V* is the vertex set of road segments with order Ν=|*V*|, *E* is the edge set of connectivity between road segments, and **A** is a Ν × Ν adjacency matrix that captures how the directed edges are connected.

Attributes of a road segment include static spatial geographic ones as ID, length, direction, and so on and a dynamic one, the speed of vehicle as a function of time.

Several feature tensors of *𝒢* are defined based on the above attributes. They are **F** ∈ ℝ^*N*× *M*× *J*^ for original geographic features, its time *t* variant **F**^*t*^ ∈ ℝ^*N*×*M*^, and static variant **F**_*s*_ ∈ ℝ^*N*×(*M* − 1)^. Correspondingly, after representation learning, these are feature tensor **S** ∈ ℝ^*N*×*D*×*J*^, static feature matrix **S** ∈ ℝ^*N*×*D*×*J*^, and dynamic feature matrix. Here *M, J, D* are the numbers of attributes of the road segment, time steps of data available, and features of the road segment after spatial representation learning, respectively.

**Definition 2 .**

(path and trajectory). A path is the sequence of road segments Ρ=〈*v*_1_, *v*_2_,…, *v*_*i*_,…, *v*_*j*_,…, *v*_*n*_〉, with |Ρ|=*n* and 1 ≤ *i* ≤ *j* ≤ *n*.

**Definition 3 .**

(traffic condition). The traffic condition ∁ ∈ ℝ^*N*×*D*×*K*^ fuses the spatial-temporal correlations and auxiliary data feature.

### 3.2. Problem Statement

*Problem Definition*. For a given path *p* and a departure time ts, a travel time query is to be performed. A multitask learning framework called DRTTE is proposed, which can return the travel time *t*_*i*_ for road segment *v*_*i*_ and *t*_en_ for the entire given path simultaneously.

*Subproblem Definition*. Prediction of traffic condition is a subproblem of TTE of each road segment and hence is carried out along with the prediction of spatial-temporal features. The kernel of the feature prediction is spatial-temporal correlation st on the object road segment. For the time series sequence st, its prediction is to get values of **K** future time steps based on the given values of **J** time steps as stated below:

(1) $$\begin{array}{c} st^{t+1}\text{,}\ldots \text{, }st^{t+K}=ℱ\left(G;\;\left(F^{t-J},\ldots ,F\text{t}\right)\right), \end{array}$$

where **F**^*t*^ is the observation feature matrix at time *t* on the object road segment. Spatial-temporal features **st**^*t* + 1^,…, **st**^*t* + *K*^ are from the dynamic feature matrix **F**^*t*^ of the past ***J*** time steps in the time sequence.

Path travel time *t*_en_ depends on path length and path speed_en_. The speed_en_ depends on traffic conditions **C** and **S**_*s*_ defined previously.

## 4. Methodology

To solve the TTE problem defined, a multitask learning framework is proposed, which consists of three major modules, namely, traffic condition module, speed module, and travel time module.  Figure 1 shows the logic structure of the framework. During the training phase, features of traffic condition **C** and speed **sp** are effectively extracted. Also, during the test phase, *t*_en_ is estimated for the given **p** and *ts*. The three kernel modules are specified below. Their inputs and outputs are detailed in Table 1.

### 4.1. Traffic Condition Module

As shown in Table 1, with original feature matrix **F**_*s*_ and adjacency matrix **A**, static spatial geographic representation of the road segments is captured as **S**_*s*_. Similarly, from **F**^*t*^ and **A**, the dynamic feature **S**^*t*^ can be captured, resulting in **st**, the spatial-temporal representation of road segments over time. Traffic condition **C**, as the core of the framework, is then obtained via fusion of auxiliary feature (e.g., weather) and **st**.

#### 4.1.1. Spatial Feature Capturing

Acquiring the traffic condition **C** is a key issue in TTE. A road segment traffic condition module is designed for its learning using adjacency matrix **A** and other feature matrices. Note that local characters of the road network are missing in the original matrices. To fix this, a convolution is used to obtain the spatial characteristics with structural information of road segments. However, due to the nature of nonregular grid of the road network data, the intricate topological structure of the road network and the spatial dependency of the road segment cannot be obtained by traditional convolution neural network (CNN).

Instead, the graph convolution network (GCN) [20] is adopted for this purpose, using a line transformation after convolution with its surrounding road segments. With a filter in spectral domain, the topology structure of the road network is captured simultaneously. Also, the spatial dependence at fixed time slice can be learned. Graph convolutional filters are used to extract the local features shared by topologically adjacent elements in graph *G*. It is seen that with GCN filters, the input stochastic weights can be “propagated” to adjacent and correlated edges during convolutions via road network topology.

Hence, capturing both static and dynamic spatial features is done via the GCN model from corresponding feature matrices of road segments, i.e., **S**_*s*_ from **F**_*s*_ and **S**^*t*^ from **F**^*t*^. Mathematically, they can be described as

(2) $$\begin{array}{c} S_{s}=\text{GCN}\left(F_{s},A\right)=\sigma \left({\dot{\text{A}}\text{F}}_{s}\text{W}\right),\\ S^{t}=\text{GCN}\left(F^{t},A\right)=\sigma \left({\dot{\text{A}}\text{F}}^{t}\text{W}\right), \end{array}$$

where $\dot{A}={\hat{D}}^{-1/2}\hat{A}{\hat{D}}^{-1/2}$ denotes the graph convolution filter, $\hat{A}=A+I_{N}$ is a matrix with self-connection structure, $\hat{D}=\sum_{j}{\hat{A}}_{ij}$ is a degree matrix, **W** is the weight matrix, and *σ*(·) represents the activation function. In Table 1, **s**_**s**_ is the row of **S**_**s**_ and denotes the learned static spatial vector for the road segment; **s**^**t**^ is the row of **S**^**t**^ and denotes the learned dynamic spatial vector for the road segment.

#### 4.1.2. Spatial-Temporal Feature Prediction

The temporal feature is another key issue in spatial-temporal correlation on each road segment. The collection forms a sequence data, which can be generally processed by the widely used recurrent neural network (RNN) that is most widely used for processing sequence data. However, the traditional RNN has limitations for long-term prediction because of the gradient vanishing and gradient explosion. The above problem has been addressed by long short-term memory (LSTM) and gated recurrent unit (GRU) models, which are designed according to the basic principle that the gated mechanism is used to memorize as much long-term information as possible. LSTM takes a longer time to train because of its complex structure. Compared with GRU, LSTM takes a longer time to train because of its complex structure and more parameters. The mathematical formulation is

(3) $$\begin{array}{c} u^{t+1}=\sigma \left(W_{u}\cdot \left[s^{t}\left[t+1\right],st\left[t\right]\right]+b_{u}\right),\\ r^{t+1}=\sigma \left(W_{r}\cdot \left[s^{t}\left[t+1\right],st\left[t\right]\right]+b_{r}\right),\\ c^{t+1}=\text{tan}h\left(W_{c}\cdot \left[s^{t}\left[t+1\right],\left(r^{t}*st\left[t\right]\right)\right]+b_{c}\right),\\ st\left[t+1\right]=u^{t}*st\left[t\right]+\left(1-u^{t+1}\right)*c^{t+1}, \end{array}$$

where *σ*(·) is an active function defined as *σ*(*x*)=(1+exp(−*x*))^−1^, **W**_*u*_, **W**_*r*_, **W**_*c*_ are weights, *b*_*u*_, *b*_*r*_, *b*_*c*_ are parameters, operator [,] represents vector concatenation, and *∗* denotes matrix multiplication.

Consequently, the GRU model is opted for temporal information processing. The spatial-temporal feature **st** at time *t* + *K* in the object road segment is predicted by a sequence of GRU cells, with the dynamic spatial feature vector **s**^*t*^ at time *t* as input.

The spatial-temporal feature **st** obtained from above can be fused with auxiliary data (such as weather **w**) to get the traffic condition **C**=[**st**, **w**], where [,] is again the concatenation operator. **C** plays a key role in the remaining modules.

### 4.2. Speed Module

The purpose of this speed module is to learn the speed on road segments in the next *K* time steps. They are known to be highly dependent on the traffic condition. Hence, **C** is taken as an influence factor of the speed feature **sp** on a single road segment at time step *t* + 1, as shown in (4). The other factor is the static spatial feature

(4) $$\begin{array}{c} sp^{t+1}=\text{LSTM}\left(C,S_{s},sp^{t};\theta_{b}\right), \end{array}$$

where *θ*_*b*_ is a parameter for LSTM.

Moreover, the connectivity nature of the road network implies that along the whole path speeds of road segments are related, especially for those adjacent segments. This higher level of dependency indicates that another update to the speed feature of the current road segment by its neighboring road segments at the time *t* + 1 is necessary.

To handle this, a graph convolution known as graph attention network (GAT) [21] is adapted to combine information about the neighbors of the object road segment. We embed the traffic from the road segment component into the path component using the GAT with time to get the traffic in the next time step along the path. The key idea is to weight the features of the neighbors using an attention mechanism. The attention coefficients from the GAT shows the level of dependency between road segments. The weight is the level of influence of neighbors on the target road segment. For target road segment *ν*_*j*_ with |*𝒩*(*j*)| neighboring road segments, the graph has |*𝒩*(*j*)| + 1$ nodes. Features of the object road segment and its neighbors are combined. The dependency of the target road segment can be represented by the *a*_*ik*_^*ts*^ using GAT. Finally, the new speed on the target road segment *𝒱*_*i*_ at next time step *ts* *+* *t* is combined by the activation function *σ*, as shown in Algorithm 1.

In (5), function **f**(·) applies the LeakReLU nonlinearity (with negative input slope = *α*0.1). When expanded, the coefficients computed by the attention mechanism can be expressed as

(5) $$\begin{array}{c} \alpha_{jk}^{ts}=\frac{\text{exp}\left(f\left(sp_{j}^{ts},sp_{k}^{ts}\right)\right)}{\sum_{i\in N\left(j\right)\cup j}\text{exp}\left(\text{f}\left(sp_{j}^{ts},sp_{i}^{ts}\right)\right)}, \end{array}$$

where **sp**_*j*_^*ts*^ is the representation speed of road segment *v*_*j*_ at time *ts*. The traffic condition is effected by the time which is the daily periodic. Intuitively, *α*_*jk*_^*ts*^ is the level of dependency or weight of road segment *v*_*k*_ on road segment *v*_*j*_.

The above procedure for speed representation on the path is implemented in Algorithm 1. There are two major steps. The first (in lines 7–11) captures the correlation to the object road segments and their neighbor road segments. Also, the second (in line 12) updates the speed of the object road in the next time step.

### 4.3. Travel Time Module

Travel time on a road segment finally depends on its length and travel speed. Here only speed needs to be calculated since length is fixed. Based on the multitask learning framework depicted in Figure 1, speed can be derived from the feature of speed $\hat{sp}$ learned from the previous two modules. This leads to travel time estimation of road segments and the entire path with $\hat{sp_{i}}$ and $\hat{sp_{en}}$.

To achieve this, $\hat{sp_{i}}$ on road segment *v*_*i*_ is designed to go through fully connected layers, resulting in the mapped scalar *speed*. Here a two-layer model instead of the traditional **LSTM** model is adopted due to its better prediction.

Speed feature **sp**_*en*_ for the entire path is a comprehensive quantity over **sp**_*i*_ for each road segment. A simple way to accomplish this is to use the mean pooling or max pooling, i.e., ${\hat{sp}}_{\text{mean}}=1/n\sum_{i=1}^{n}\hat{sp_{i}}$. However, the largely uneven speed features on each road segment lead to significant error of the above pooling. To improve, the equal-weight 1/*n* can be replaced by a set of specially designed weights, as in the following attention mechanism.

${\hat{sp}}_{att}=\sum_{i=1}^{n}\alpha_{i}\hat{sp_{i}}$ , where *α*_*i*_=exp(**sp**_**i**_)/∑exp(**sp**_**i**_) is the normalized weight for the *i*-th road segment. The resulting ${\hat{sp}}_{att}$ is then fed to residual fully connected blocks that train a very deep neural network [22]. Based on the above result, ${\hat{sp}}_{en}$ is finally obtained via a MLP simple neural network model.

## 5. Experiments

### 5.1. Experiment Settings

Effectiveness and overall performance of the DRTTE model are evaluated on two large-scale real-world taxi datasets, namely *Harbin* and *Chengdu*. For convenience, continuous road networks are segmented into discrete parts, and two-dimensional GPS data are transformed accordingly along with road segment ID by map matching algorithm [23]. We adopt Adam algorithm [24] optimization to train the parameters of the model. The learning rate is 0.001. We select the best models by 3-fold cross-validation.

#### 5.1.1. Evaluation Metrics

The evaluation metrics we adopt include mean absolute percentage error (MAPE), root mean squared error (RMSE), and mean absolute error (MAE). MAPE compares the estimation value to the percentage of the ground-truth value, while RMSE and MAE are the gaps between estimation and true values.

### 5.2. Comparisons with Baselines

Results in performance of DRTTE are compared against the baseline methods including ARIMA, TEMP [25], and DeepTTE [6].  Table 2 shows the details. It is seen that ARIMA is the lowest performing method. TEMP gives medium performance and cannot cope with the complicated traffic conditions either. TEMEP and DeepTTE work better than ARIMA, but DRTTE outperforms them significantly on the two datasets.

The reason is twofold. Firstly, static and dynamic spatial information can be obtained by DRTTE using graph convolution operations. Secondly, the dependency among the road segments with road properties can be captured by graph attention network. These innovations help preserve the spatial-temporal characteristics of the traffic condition and the relationship between the road segments.

### 5.3. Efficiency of Different Components

There are four significant components in DRTTE, i.e., LSTM, GCN, GRU, and GAT. Building upon the base model LSTM, other components are selectively combined, resulting in four models with new features potentially in an order of higher-level accuracy.

1. “LSTM”: multitask learning without information of road segments and road network characters.
2. “LSTM + GCN + GRU”: with spatial-temporal information of the road segments.
3. “LSTM + GCN + GRU + GAT”: with dependency between road segments.
4. “LSTM + GCN + GRU + GAT + attention”(DRTTE): with attention mechanism in the multitask layer.

Their effectiveness and efficiency are measured using the set of metrics, with results given in Table 3. Several observations can be made. Firstly, “LSTM” exhibits the lowest performance. Secondly, “LSTM + GCN + GRU” is comparable to DeepTTE in performance due to their similar structures of model framework. However, the spatial-temporal feature time series prediction of each road segment is missing in DeepTTE. This limits its capacity in accurate travel time estimation of the entire path. Thirdly, “LSTM + GCN + GRU + GAT” performs better than DeepTTE since the latter lacks the dependency of the speed of the adjacent road segment. Lastly, DRTTE performs even better than “LSTM + GCN + GRU + GAT” with the help of attention mechanism.

The above comparisons show that DRTTE is the best in the set of methods built on LSTM. It addresses spatial-temporal feature time series prediction of each road and dependency of the speed of the adjacent road segment, enabling it to estimate travel time in a more efficient way with higher accuracy.

### 5.4. Travel Times and Distance Patterns

Effects of travel distance to MAPE and MAE are depicted in Figure 2. The calculations are based on 9,870 road segments randomly selected from the validation datasets. Figure 2 shows that with increasing length of path, both DeepTTE and DRTTE see loss of accuracy in different degrees. This is natural and expected since uncertainty of traffic condition increases with the length of path, resulting in performance degradation for any model inevitably. However, it is noted that the percentage estimation error of DRTTE is well controlled (13%∼20%) for intermediate lengths (2∼7 km), while this range for DeepTTE is (17%∼ 30%). Also, in the field test, the MAE of DRTTE is controlled in around 2.4 minutes, while for DeepTTE, it is around 3 minutes. This shows that DRTTE gains around 20%∼30% in accuracy on average compared to DeepTTE and is less sensitive to distance.

Results of MAPE and MAE with epoch amounts of “20, 40, 60, 80, and 100” are depicted in Figure 3. It is seen that a higher epoch reduces the MAPE from (Chengdu 50.75%, Harbin 42.23%) to (Chengdu 13.91%, Harbin 11.64%) and reduces the MAE from (Chengdu 320.75 s, Harbin 280.23 s) to (Chengdu 155.71 s, Harbin 136.29 s). These results demonstrate the effectiveness of epoch for accuracy improvement of travel time estimation.

### 5.5. Effects of Kernel Size

Figure 4 shows the effects of kernel size of the graph convolutional operation. It is seen that the MAPE, MRSE, and MAE have the same trend, and the best results are obtained when the kernel size is intermediate. When the kernel size is less than 4, spatial correlation cannot be captured entirely, but when it is greater than 4, more unnecessary information is captured that damages the true correlation between road segments.

## 6. Conclusion

In this work, we proposed a novel multitask learning framework DRTTE to explore the effect of spatial-temporal correlation of the traffic to travel time estimation, considering traffic conditions and dependency relationship of road segments. The effectiveness and efficiency of DRTTE are validated based on experiments of two real taxi trajectory datasets. Our findings show that the proposed framework outperforms the existing methods with higher level of accuracy. More importantly, it is demonstrated that the spatial features have significant effects to travel time estimation. Future work will focus on federated learning for travel time estimation to prevent privacy leaking.

## Figures and Tables

**Figure 1:** The architecture of dependent relationship travel time estimation (DRTTE).

**Figure 2:** Effects of travel distance to MAPE and MAE.

**Figure 3:** Effects of epoch.

**Figure 4:** Effects of kernel size to MAPE, RMSE, and MAE.

**Algorithm 1:** The dependency between road segments along the path.

**Table 1:** The input and output variables of the modules.

	Traffic module			Speed module			Travel time module	
Input	**A**, **F**_*s*_	**A**, **F**^*t*^	**S** ^*t*^	**st**, **w**	**S**_*s*_, **C**	**sp**	**s**ˆ**p**	Speed, length
Model	GCN	GCN	GRU			GAT	Multitask learning	
Output	**S**_*s*_	**S** ^*t*^	**st**	**C**	**sp**	**s**ˆ**p**	Speed	*t*

**Table 2:** Performance comparison with baselines.

	Chengdu			Harbin		
	MAPE (%)	RMSE (sec)	MAE (sec)	MAPE (%)	RMSE (sec)	MAE (sec)
ARIMA	35.49	444.42	357.22	32.32	413.62	310.47
SimpleTTE/TEMP	26.45	324.18	213	22.75	314.08	193.61
DeepTTE	19.37	289.51	191.26	17.61	267.04	164.23
DRTTE (this work)	**13.91**	**252.32**	**155.71**	**11.64**	**242.7**	**136.29**

**Table 3:** Efficiency of different components.

	Chengdu			Harbin		
	MAPE (%)	RMSE (sec)	MAE (sec)	MAPE (%)	RMSE (sec)	MAE (sec)
LSTM for multitask learning	30.14	312.84	241.09	29.47	309.64	232.76
LSTM + GCN + GRU	19.25	286.02	207.98	18.78	262.65	183.91
LSTM + GCN + GRU + GAT	16.48	276.06	188.18	15.16	230.22	167.56
DRTTE (this work)	13.91	252.32	155.71	11.64	242.7	136.29

## Data Availability

The data underlying the results presented in the study are included within the article.
